This article has been retracted.

# Identification of C-T novel polymorphism in 3^rd^ exon of *OsSPL14* gene governing seed sequence in rice

**DOI:** 10.1371/journal.pone.0264478

**Published:** 2022-03-14

**Authors:** Muhammad Salah ud Din, Xiukang Wang, Salman Alamery, Sajid Fiaz, Haroon Rasheed, Muhammad Abid Khan, Shahid Ullah Khan, Sumbul Saeed, Niaz Ali, Kalim Ullah Marwat, Kotb Attia, Itoh Kimiko, Shabir Hussain Wani

**Affiliations:** 1 Department of Botany, Hazara University, Mansehra, Khyber Pakhtunkhwa, Pakistan; 2 College of Life Sciences, Yan’an University, Yan’an, Shaanxi, China; 3 Department of Biochemistry, College of Science, King Saud University, Riyadh, Saudi Arabia; 4 Department of Plant Breeding and Genetics, The University of Haripur, Haripur, Pakistan; 5 Department of Botany, University of Science and Technology Bannu, Khyber Pakhtunkhwa, Pakistan; 6 Institute of Nuclear Agriculture Sciences, College of Agriculture and Biotechnology, Zhejiang University, Zijingang Campus, Hangzhou, PR China; 7 Department of Biochemistry, Women Medical and Dental College Abbotabd, Khyber Pakhtunkhwa, Pakistan; 8 College of Plant Sciences and Technology, Huazhong Agricultural University, Wuhan, P.R. China; 9 Department of Zoology, Kohat university of Science and Technology, Kohat, Khyber Pakhtunkhwa; 10 Institute of Science and Technology, Niigata University, Nishi-ku, Niigata, Japan; 11 Mountain Research Center for Field Crops, Khudwani, Sher-e-Kashmir University of Agricultural Sciences and Technology Srinagar, Srinagar, J&K, India; University of Education Lahore, Pakistan, PAKISTAN

## Abstract

Recently food shortage has become the major flagging scenario around the globe. To resolve this challenge, there is dire need to significantly increase crop productivity per unit area. In the present study, 24 genotypes of rice were grown in pots to assess their tillering number, number of primary and secondary branches per panicle, number of grains per panicle, number of grains per plant, and grain yield, respectively. In addition, the potential function of miR156 was analyzed, regulating seed sequence in rice. Furthermore, *OsSPL14* gene for miR156 was sequenced to identify additional mutations within studied region. The results demonstrated Bas-370 and L-77 showed highest and lowest tillers, respectively. Bas-370, Rachna basmati, Bas-2000, and Kashmir Basmati showed high panicle branches whereas, L-77, L-46, Dilrosh, L-48, and L-20 displayed lowest panicle branches. Bas-370 and four other studied accessions contained C allele whereas, L-77 and 18 other investigated accessions had heterozygous (C and T) alleles in their promoter region. C-T allelic mutation was found in 3^rd^ exon of the *OsSPL14* gene. The sequence analysis of 12 accessions revealed a novel mutation (C-T) present ~2bp upstream and substitution of C-A allele. However, no significant correlation for novel mutation was found for tillering and panicle branches in studied rice accessions. Taken together present results suggested novel insight into the binding of miR156 to detected mutation found in 3^rd^ exon of the *OsSPL14* gene. Nevertheless, L-77, L-46, Dilrosh, L-48, and L-20 could be used as potential breeding resource for improving panicle architecture contributing yield improvement of rice crop.

## Introduction

Rice (*Oryza sativa* L.) is among essential monocotyledonous plants belongs to family *Poaceae* and consumed by more than 50% of people around the world. Global food security is becoming a serious challenge for rapidly growing human population owing to negative environmental conditions caused by climate change [1, 2]. Therefore, it is important to accelerate the productivity of crops through breeding superior varieties. Among varipus attributes, tillering is considered an essential characteristic to determine rice yield because its significant correlation with cereal production [3]. Plants with high tillers might be useful for adapting to diverse environmental condition however, low tillers severely influence extreme stress conditions [4]. In Pakistan, rice has become next staple food after wheat, and a source of foreign earning through export. From the last several decades, agriculture system of Pakistan has faced severe challenges [5]. In Punjab Gujranwala, Sheikh Khupura, and Sialkot are the main rice producing areas whereas, few districts of Punjab and Sindh are less rice cultivated areas [6]. On global scale, over three billion Asian people meet their caloric requirements from rice [7]. In addition, it has been estimated that from 2001 to 2025, global demand for rice production is expected to increased by 25%, and an annual increase of 5.9 metric tons is required to achieve. However, to meet caloric demand for ever-increasing human population, the Food and Agriculture Association of the United States forecasted that by 2050 the rice demand will exceed by 524 metric tons, and productivity of rice is estimated to increase by 2 metric tons per year compared to current rice production [8].

During the last three years, rice production has reached to a record level. During 1940–1960s, green revolution led to an expansion in creation of agro-based industry especially in devolving countries, primarily through progress in research and innovation [9]. The new rice varieties, grown on irrigated land in half of the world’s crops, contribute almost three-quarters to total rice production. Fifteen countries are contributing 90% of the world’s rice production [10] whereas, only China and India account for 50% of rice cultivation.

Tillering begins around 40 days after planting and can last up to 120 days. It is a physiological process of continuous underground branching of compact node joints of the primary shoot. Tillering gives the crop the necessary number of stalks required for a good production. Tillers emerging in this way from nodes in the main culm are called primary tillers. These emerge all through the vegetative growth phase, but stop when plants reach panicle initiation (the starting point of the reproductive phase). These tillers emerge and branch out from the base of the plant. After panicle initiation, tillers may continue to emerge from preexisting tillers, filling out the space among plants. These tillers are called secondary tillers. Plant hormones such as auxin, cytokinin [2, 11], and strigolactones [12, 13] control axillary bud outgrowths. The main *PROTEIN BINDING TO THE SOUAMOSA 14 PROMOTER* (*OsSPL14*) is regulated by micro RNA Osmi156, the improved level of transcription and protein *OsSPL14* results in an IPA phenotype and greater cereal productivity [2, 14]. The QTL *WFP (WEALTHY FARMER’S PANICLE)* encoding *OsSPL14* contrarily manages the numbers of tillers in the asexual phase and exactly switches the quantity of rachis in the reformative period. The greater manifestation of *OsSPL14* in young panicles stretched panicle wafting and grain number per panicle, contribute increase yield of rice [15, 16].

Lower DNA methylation on this allele increases the transcription frequency of *OsSPL14*, which leads to a high number of grains per panicle. There is a substitution of nucleotides C to T from the start codon in the promoter region at a distance of 4.2 kb. Nucleotide C is a target methylation site; nucleotide T avoids methylation with a higher manifestation of *OsSPL14* [14, 17]. Another allele with synonymous substitution of C for A at 3^rd^ exon of *OsSPL14*, a target site (complementary site in the coding region) of OsmiR156. Previous studies reported that OsmiR156 targets approximately 11 *OsSPL* genes. OsmiR156 cleaves the *OsSPL14* mRNA, if *OsSPL14* carries the wild-type nucleotide C at target site.

OsmiR156 is strongly expressed in vegetative shoots, leaves, and the tip but is suppressed in the early stages of panicle development [14, 18]. Introduction of the high-efficiency *OsPL14WFP* allele to the standard Nipponbare rice variety leading to increased rice production [14]. In-plant architecture, tillering is an important component that increases rice yield and crop components. As a complex agronomic element, a rice plant’s grain yield can be duplicated by three-segment attributes: number of panicles per plant, number of grains per panicle, and grain weight. The quantity of panicles relies upon the plant’s capacity to deliver tillers (tillering limit), comprising essential, auxiliary, and tertiary tillers. The size of the grain controls the total grian weight. It is indicated by its three measurements (length, width, and thickness) and the level of substantial [2, 11]. The genes *EHD1* and *HD1* involve in photoperiodic controlling and ultimately timmering. An expanded level of articulation of *HD3A* and *RFT1* reduces the number of essential branches per piston in the line that consolidates *HD1* and *EHD1* [19]. *HD1* builds up the number of spikelets per piston and grain by suffocating the *Hd3a* joint and shifting the date. Here we reported the genetic and molecular analysis of the *OsSPL14* gene and proposed some functional features of rice genotypes for the evaluation of *OsSPL14* in panicle branching and the regulation of grain yield in rice. Hence our proposed result may suggested that the new mutation in *OsSPL14* can play a significant and potential role in tillering, and grain yield in rice, respectively.

## Material and methods

The study was conducted at the Department of Botany, University of Science and Technology, Bannu during year 2018. A total of 24 rice genotypes and varieties were investigated in current study (S1 Table). For convenience, all these selected genotypes and varieties are referred to as lines in subsequent text. Seeds of the selected germplasm were obtained from NARC, Islamabad, Pakistan. Two lines Basmati-370 and Line-77 were used as check in present investigation and grown under CRD (completely randomized design).

### Germination of rice seedlings

Seed of the selected 24 rice genotypes (Table 1) were grown in replicates following CRD, mature paddy seeds were harvested from each accession.

**Table 1:** Evaluation of important yield contributing traits within selected germplasm.

Accession	NT	NG	BP	NGP	SBP	GW (kg)
**BAS-370**	27.66^A^	187.67^A^	11.667^AB^	3753.3^A^	6.3333^BCDE^	0.0369^ABCD^
**RACHNA Basmati**	27.00^AB^	123.67^GH^	11.333^ABC^	2398.7^B^	7.3333^ABC^	0.0653^A^
**Bas-2000**	25.000^BC^	172.00^B^	12.333^A^	2486.7^B^	8.0000^A^	0.0510^ABC^
**Kashmir Basmati**	24.667^BC^	174.00^B^	12.000^AB^	1740.0^C^	6.6667^ABCD^	0.0387^ABCD^
**Bas-385**	23.333^CD^	178.33^B^	12.667^A^	2445.7^B^	7.6667^AB^	0.0503^ABC^
**Fakher-e-Malakand**	23.000^CDE^	160.33^C^	11.667^AB^	1603.3^CD^	5.6667^DEFG^	0.0357^ABCD^
**Swat II**	22.000^DEF^	142.33^D^	10.667^BCD^	1406.3^DEF^	5.0000^EFGH^	0.0327^ABCD^
**IR9**	21.000^DEFG^	89.67^L^	8.667^EF^	1224.7^F^	5.0000^EFGH^	0.0407^ABCD^
**L-146**	20.667^EFGH^	118.67^H^	8.000^FG^	1186.7^F^	4.3333^GH^	0.0263^BCD^
**NPT 22**	20.000^FGH^	137.67^DE^	8.333^FG^	1522.7^CDE^	5.0000^EFGH^	0.0370^ABCD^
**KSK-133**	19.000^GH^	159.33^C^	12.333^ABC^	660.7^C^	6.6667^ABCD^	0.0397^ABCD^
**SWAT-I**	19.000^GH^	128.67^FG^	8.667^EF^	1286.7^E^	5.6667^DEFG^	0.0340^ABCD^
**Bas p-s 2**	18.338^H^	133.33^EF^	7.000^CDE^	1333.3^EF^	6.0000^CDEF^	0.0333^ABCD^
**L-31**	15.667^I^	96.33^JKL^	6.333^H^	775.3^G^	3.6667^H^	0.0183^CD^
**Muskan**	15.667^I^	127.00^FGH^	8.667^EF^	1270.0^G^	4.0000^H^	0.0310^ABCD^
**Malkhar-346**	15.333^I^	103.00^IJK^	9.333^DEF^	793.0^G^	5.6667^DEFG^	0.0237^CD^
**L-134**	14.000^IJ^	108.00^I^	8.667^EF^	756.0^G^	5.0000^EFGH^	0.0187^CD^
**KSK-434**	13.667^IJK^	90.00^L^	10.000^CDE^	660.7^G^	6.0000^CDEF^	0.0163^CD^
**P-5**	13.333^IJK^	106.33^I^	7.000^GH^	744.3^G^	3.6667^H^	0.0150^CD^
**L-20**	12.667^JKL^	92.67^L^	8.333^FG^	588.0^GH^	4.3333^GH^	0.0433^ABCD^
**L-48**	12.667^JKL^	94.33^KL^	8.000^FG^	660.3^G^	5.6667^DEFG^	0.0170^CD^
**Dilrosh**	12.333^JKL^	104.67^IJ^	8.667^EF^	625.0^GH^	5.0000^EFGH^	0.0180^CD^
**L-46**	11.333^KL^	96.00^JKL^	8.000^FG^	544.3^GH^	4.6667^FGH^	0.0617^AB^
**Line-77**	10.666^L^	66.33^M^	8.000^FG^	376.3^H^	5.0000^EFGH^	0.0083^D^
**Grand mean**	18.250	124.60	9.5278	1328.6	5.5000	0.0330
**Maximum**	27.667	187.67	12.667	3753.3	8.0000	0.0653
**Minimum**	10.667	66.33	6.333	376.3	3.6667	0.0083
**CV%**	8.67	4.33	8.77	11.93	17.60	66.85

NT = Number of tillers, NG = Number of grains per panicle, PBP = Branches per panicle, NGP = Number of grains per plant, SBP = Secondary branches per panicle, GW = Grain weight.

### Morphological characterization

The plants were scored for six morphological characters based on International Rice Research Institute’s descriptor, Manila Philippines [18]. Total number of tillers was recorded by counting total number of tillers from randomly selected three plants and taken their average value. Number of filled grains in a single panicle from three plants was calculated, and their average value was calculated. Number of grains per plant were calculated selecting three random plants form each line. Thousand-grain weight was recorded using a digital balance. Branches per panicle were recorded selecting three plants from each genotype and averaged. Number of secondary branches per panicle was counted from three randomly selected plants of each line and averaged.

### Molecular characterization

DNA extraction was performed from young leaf tissues via modified CTAB method [20]. To validate the expected DNA fragment gel electrophoresis was performed. During current study, seven primers were used along with four pairs of markers to detect the SNPs C/T and C/A in third exon of *OsPL14* gene (S2 Table). These primers were selected from [13] to amplify and sequencing of *OsPL14* gene promoter.

### PCR amplification and nucleotide sequencing

PCR amplification was carried out using PROMEGA kit Madison Company USA. PCR master mix was prepared for a total of 24 samples having18 μl for each sample. The individual sample reaction contains 12.24μl of water 2Mm MgCl_2_, taq buffer of 0.4 μl. 0.2 μl for each forward and reverse primer of 20Mm 0.4 of DNTPS and 0.16 of tag polymerase. Template DNA of 2 μl corresponding to 100ng was used. PCR conditions were set for 40 cycles set at 94°C for 2min, followed by 30 seconds 94°C, 30 sec on 55 °C and 72°C for 30 sec, and final extension of 72°C for 10 min. Once the desired PCR products were confirmed, template DNA was sent to tsingke Biotechnology Company, China for sequencing of seed sequence for miR156 third exon of *OsSPL14* gene to detect potential mutation.

### Statistical analysis

The morphological data was analysed using, statistic 8.1 [19]. The sequencing result was first aligned to reference rice gene *OsPL14* (838692 gene ID) available at NCBI (https://www.ncbi.nlm.nih.gov/). Crustal W multiple alignment tools were used to carried out multiple sequence alignment to identify potential SNP_S_. BLAST and I-TASSER were utilized to analyze the effect of SNPs for amino acid substitution on protein structure. The PDB file of the selected model was further subject to ERRAT-2 program to generate overall quality factor for OsSPL14 protein. Estimated RMSD and TM score and respective was run in ERRAT-2 to generate an overall quality score.

## Results

### Morphological traits results

Morphological evaluation of genotypes showed highest number of tillers for Basmati 370, the lowest was recorded for Line 77. Similarly, the highest grains per panicale were recorded for basmati 370 whereas, Line 77 showed the lowest number of grains per panicale. The highest number of panicles per branches were recorded for Basmati 385, whereas, the lowest were observed in Line 33. Highest number of grains per plant were recorded for Basmati 370 whereas, lowest grains per plant were recorded for Line 77. In addition, Basmati 200 had the highest secondary branches per panicle, while P-5 had the lowest secondary branches per panicle.

The grain weight was also accounted for among the investigated germplasm, the highest grain weight was recorded for Rachna, while the lowest was recorded for Line 77. The maximum value for the variation coefficient was recorded for grain weight, and the number of grains per panicle and revealed the lowest. Importantly, all traits showed significance for scored traits, as represented in (Table 1).

### Correlations among important yield contributing traits

The association of various traits is essential to collect information for quality and yield related traits in rice. To understand the magnitude and nature of the association between the investigated traits i.e., number of tillers per plant, number of grains per panicle, primary branches per panicle, number of grains per plant, secondary branch per panicle, and grain weight were subjected to pearson’s correlation, results are shown in (Table 2). Pearson’s correlation revealed that the number of tillers per plant showed a significant correlation with the number of grains per plant, followed by several grains per panicle. The tillers per plant also showed a strong and highly significant correlation of 0.7620, 0.6313, and 0.5671 with primary branches per panicle, secondary branches per panicle, and grain weight, respectively.

**Table 2:** Pearson correlation among the six yield attributing traits.

	**NT**	**NG**	**PBP**	**NGP**	**SBP**
**NG**	0.8120**				
**PBP**	0.7620**	0.8139**			
**NGP**	0.8987**	0.8539**	0.7629**		
**SBP**	0.6313**	0.6269**	0.8713**	0.6691**	
**GW**	0.5671**	0.4649*	0.5261**	0.5446**	0.5066*

NT = Number of tillers, NG = Number of grains per panicle, PBP = Branches per panicle, NGP = Number of grains per plant, SBP = Secondary branches per panicle, GW = Grain weight

*significant at P<0.05

** Significant at P<0.01

Furthermore, the number of grains per panicle showed a significant correlation with number of grains per plant followed by primary branches per panicle and secondary branches per panicle. A significant correlation was recorded between the number of grains per panicle and grain weight. Primary branches per panicle also showed a highly significant correlation with secondary branches per panicle, followed by the number of grains per plant. The number of primary branches per panicle also revealed a highly significant correlation with the grain weight. The number of grains per plant also manifested a highly significant correlation with secondary branches per panicle, followed by grain weight. Nonetheless, a significant correlation was recorded between secondary branches per panicle and grain weight.

### Molecular genotyping

PCR amplification of *SPL14-04* regains for C-T allele genotyping. Highly quality DNA extracted was used for PCR amplification. The *SPL14-14* region was amplified with CR and TR primers that resulted in 267bp amplicons (Fig 1, Table 3). Out of the 24 rice lines and varieties used, 5 had C type allele, whereas 19 contain heterozygous with a C-T allele. The reference genome of *SPL14* undergo both symmetric and asymmetric methylation therefore, C allele is a target nucleotide for methylation in the promoter region of the *OsSPL14* gene, which regulates the expression level of a gene. The C-T substitution prevents methylation and may interfere with the transcription of gene through epigenetic phenomena. Basmati 370, IR9, Malkhar-346, Line 20, and Line 31 carry wild type C allele while Rachna basmati, Line 77, KSK 434, Dilrosh, swat I, Kashmir basmati, Line 46, Line 48, Line 146, Basmati 385, NPT 22, Basmati 200, KSK 133, P-5, Muskan, Swat II, Malakand, P.S 2 carry heterozygous C-T Allele.

**Fig 1:** Depicted accession in study for C -T allele.

**Table 3:** List of rice germplasm carrying C or T allele.

S. No	Land races	Allele	S. No	Land races	Allele
**1**	Rachna basmati	C	13	Line 134	C-T
**2**	Basmati 370	C	14	Line 48	C-T
**3**	IR9	C	15	Line 146	C-T
**4**	L-77	C	16	Basmati 385	C-T
**5**	KSK 434	C	17	NPT 22	C-T
**6**	Dilrosh	C-T	18	Basmati 200	C-T
**7**	Malkhar	C-T	19	KSK 133	C-T
**8**	Swat-I	C-T	20	P-5	C-T
**9**	Kashmir basmati	C-T	21	Muskan	C-T
**10**	L-20	C-T	22	Swat II	C-T
**11**	Line 46	C-T	23	Malakand	C-T
**12**	Line 31	C-T	24	P.S 2	C-T

### *SPL14-12* C-A allele genotyping

PCR amplification was carried out for C-A allele in fragment size of 244bp and 302bp. All the accessions carry a C allele in fragment size of 244bp. C-A allele was located on third exon of *OsSPL14*, which is the target site of OsmiRNA156. OsmiRNA156 is a free miRNA that cleaves the mRNA transcript of the *OsSPL14* gene. Rachna basmati, Basmati 370, IR9, 77, KSK 434, Dilrosh, Malkhar, Swat-I, Kashmir basmati, Line 20, Line 46, Line31, Line 134, Line 146, Basmati 385, NPT 22, Basmati 200, KSK 133, P.5, Muskan, Swat-II, P.S 2, DR 2 carried the wild type C allele (Fig 2, Table 4).

**Fig 2:** Depicted accession in study for C-A allele.

**Table 4:** List of rice germplasm C- A allele.

S. No	Land races	Allele	S. No	Land races	Allele
**1**	Rachna Basmati	C	13	L-134	C
**2**	Basmati 370	C	14	L-48	C
**3**	IR9	C	15	L-146	C
**4**	LinE-77	C	16	Basmati 385	C
**5**	KSK-434	C	17	NPT 22	C
**6**	Dilrosh	C	18	Basmati 200	C
**7**	Malkhar	C	19	KSK 133	C
**8**	Swat-I	C	20	P-5	C
**9**	Kashmir Basmati	C	21	Muskan	C
**10**	L-20	C	22	Swat II	C
**11**	L-46	C	23	Fakher-e-Malakand	C
**12**	L-31	C	24	P.S 2	C

for **C allele** 1 = Rachna Basmati, 2 = Basmati 370, 3 = IR9, 4 = 77, 5 = KSK 434, 6 = Dilrosh, 7 = Malkhar, 8 = swat-I, 9 = Kashmir Basmati, 10 = Line 20, 11 = Line 46, 12 = Line31, 13 = Line 134, 14 = 48, 15 = Line 146, 16 = Basmati 385, 17 = NPT 22, 18 = Basmati 200, 19 = KSK 133, 20 = P.5, 21 = Muskan, 22 = Swat-II, 23 = Fakher-e-Malakand, 24 = P.S 2 M = Marker

### Sequencing of *OsSPL14* for OSmiR156 target-site

The irregularity of visual correlation between tiller number per plant and the respective allele was sequenced at the 3^rd^ exon of *OsSPL14* gene, which carries OSmiR156 directed transcriptional cleavage, if any additional mutation in miRNA target site. Interestingly, the sequence result revealed a new single nucleotide polymorphism (C-T substitution) in 09 different accessions, 2bp upstream of the previous reported SNP (C-A) [14, 18] in the target seed sequence for miRNA156 (Fig 3).

**Fig 3:** Aikawa1 and ST-12 are the two control sequences along reference genome (Nipponbare).

### Analysis of protein for new mutation

The nucleotide sequence was translated using NCBI BLAST online tool which aligned translated sequence of new SNP (C-T) mutation carrying *OsPL14* revealed an amino acid substitution from alanine to valine (Fig 4). The aligned sequence showed 99% sequence homology with *SQUAMOSA PROMOTER BINDING PROTEIN-LIKE 14*. Both alanine and valine amino acids are internal, hydrophobic, and neutral.

**Fig 4:** Amino acid alignment to missense mutation indicates from alanine to valine.

To further understand the structural change in *SQUAMOSA PROMOTER BINDING PROTEIN-LIKE 14*, due novel mutation, the sequence results of both wild type and valine carrying gene were analyzed using I-TASSER that generated different models. The models chosen were based on RMSD, C-score, and TM-Score (Table 5). The best model was subjected to ERRAT2 software that predicted both sequences’ quality factor (Fig 5).

**Fig 5:** **(A)** Overall quality factor of wild type protein. **(B)** Overall quality factor of C-T substitution.

**Table 5:** Protein model score of the predicted wild and alanine to valine substitution.

Models	Evaluation Scores			Overall quality factor (ERRAT2 used)
	C-score	Estimated RMSD	Estimated TM-Score	
Wild type *OsSPL14*	-1.08	9.4+-4.6A	0.58+-0.14	62.703
Alanine to Valine change in *OsSPL14*	-0.79	8.7+-4.5A	0.61+-0.14	62.703

The Models (Fig 6A & 6B) for wild type and alanine to valine substituted *OsSPL14* gene was selected among the five predicted models for each with large decoys (cluster density) based on pairwise structural similarities. C-score quantitatively measures each models’ confidence based on the significance of threading template alignment and the structural assembly simulations’ convergence parameter. C-score ranges from -5 to 2, which signifies high confidence of the model. A model of C-score more -1.5 indicated correct global topology. In the present study, the substituted amino acid alanine to valine of OsSPL14 protein has a value of -0.79. Template Modelling Score (TM-score) compares two model structural alignment based on the amino acid residues and measures the structural homology. The TM-Score ranges from 0–1. The query substituted amino acid protein exhibited high TM-score (0.61+-14) compared to template Protein Data Bank in the present data. In Figs 5 and 6 at position 290 the substitution of amino acid from alanine to valine (Fig 5) shows the same error value as in the wild type (Fig 6A & 6B), and ERRAT2 generated the same quality factor score as for the wild type.

**Fig 6:** (A) Wild type (B) Alanine to Valine substitution. Model generated by I-TASSER.

## Discussion

Rice tillers are produced on stunted basal internode that develop freely on the main stem having adventitious root. Tillering in rice is among the major constituent of rice grain yield [20]. *OsSPL14*, *IDEAL PLANT ARCHITECTURE (IPA)*, and *WEALTHY FARMER GENE (WFP)* are major genes that tailors rice tillers and panicle branches. Regarding *OsSPL14* expression, OsmiR156 plays an essential and dual role in tillers regulation, number of panicles branching and spikelet’s development [14, 18]. This study analyzed 24 genotypes of rice accessions based on structural and molecular characterization to estimate the genetic diversity. Based on morphology, 6 traits were observed in 24 genotypes of rice. The sequence analysis showed presence of variation in the given data set among 24 genotypes i.e., Number of tillers plant, number of grains per panicle, secondary branched panicle, number of grains per plant, grain weight, as shown in (Table 1). In the present study number of tillers per plant, the number of grains per panicle, and the secondary branched panicle showed significant variation.

A highly significant correlation was observed in the number of grains per panicle with the number of grains per plant followed by primary branches per panicle and secondary branches per panicle, respectively. A significant correlation was recorded between the number of grains per panicle and grain weight. Primary branches per panicle also showed a highly significant and strong correlation with secondary branches per panicle, followed by several grains per plant. The number of tillers per plant also showed a strong and highly significant correlation of 0.7620, 0.6313, and 0.5671 with primary branches per panicle, secondary branches per panicle, and grain weight, respectively. Similarly, the same work was conducted by [21], who observed a high variation among the seven traits. Correlation coefficients between all pairs of variables used in this experiment are shown in (Table 2).

The C allele ~2.6 kb mapped on the upstream at the start codon of SPL14-04 site is an epigenetic manner. The allele-specific amplification of this heritable epigenetic allele in the promoter region revealed nineteen samples as heterozygous (C and T). Previous research reported five heterozygous alleles out of 12 in BC_2_F_2_ plants derived from a cross between PR38012 and ST-12 [17]. However, due to the heterozygosity of the allele in most of the accessions, no valid correlation was observed between the heritable epigenetic allele and the number of tillers. Micro RNA plays an essential role in regulating many target genes. In plants, miRNA inhabits many genes, while in animals, it represses translation [22–24]. OsmiR156 expression lowered at the panicle development stage [14, 18]. The *SPL* genes are regulated by microRNA miR156, and *OsSPL16* of OsmiR156 was shown to repress *OsSPL16* transcription in young panicles [25].

In previous studies, no C-A mutation was found however, the sequence analysis result revealed a new C-T mutation located at ~2bp upstream of the *OsSPL14* gene. Hexapeptide ALSLLS is a conserved motif of *SQUAMOSA PROMOTER BINDING PROTEIN-LIKE 14* [26]. However, substitution with VLSLLS in the mutant type has no negative effect on the protein as predicted by I-TASSER and ERRAT2 model. The binding of miR156 to the seed sequence of SPL-14 indicates the amount of *SQUAMOSA PROMOTER BINDING PROTEIN-LIKE 14* gene expressions. The average effect of the T allele in the seed sequence for miR156 on the number of grains per plant is the same as the wild-type allele, which suggests further insight that this new mutation (C-T) substitution did not inhibit the binding of the miR156 to the target site. Previous studies reported that microRNA imperfectly binds to seed sequence [25, 27, 28]. We also identified some lines that showed low grains per panicle, so we suggested that it might be some other genes regulating grain per panicle. Moreover, Line-20 and Line-77 carry low grains per panicle. Similarly, the grain yield per plant of Line-77, Line-20, and Line-48 also had low grain yield per plant.

## Conclusion

We identified for the first time a new C-T mutation in the third exon of the *OsSPL14* gene in rice which can play an important role in grain yield development. Mutation of *OsSPL14* in rice demonstrated the number of tillering and grain size based on phenotyping results, molecular characterization, and statistical analysis, respectively. Hence our present findings not only identified *OsSPL14* as a key regulator of grain yield but also suggest a strategy for the modification of grain yield in a wide range for the improvement in crops.

## Supporting information

S1 Table List of selected genotypes. (DOCX)

S2 Table Allele specific molecular marker used in the study. (DOCX)

S1 Raw image (DOCX)
